The article "The Efficacy of Adjuvant Targeted Therapy in Patients with Advanced Renal Cell Carcinoma: A Systematic Review and Meta-Analysis" was retracted in 2023. Reasons: unreliable results or conclusions; concerns about the data; concerns about the peer review; concerns about the citations.

# The Efficacy of Adjuvant Targeted Therapy in Patients with Advanced Renal Cell Carcinoma: A Systematic Review and Meta-Analysis

**DOI:** 10.1155/2022/7341294

**Published:** 2022-03-29

**Authors:** Wingkeung Yiu, Jie Chen, Binglin Zhao, Weiqing Zhang, Linlin Chen, Hua Liu

**Affiliations:** ^1^Urinary Surgery, The First Affiliated Hospital of Jinan University, Guangzhou, China; ^2^Nankai University, Tianjin, China; ^3^Urinary Surgery, Southern Hospital of Southern Medical University, Guangzhou, China

## Abstract

**Background:**

The aim of this systematic evaluation and meta-analysis was to analyze the efficacy and adverse effects of adjuvant targeted therapy regimens in advanced or metastatic renal cell carcinoma (RCC).

**Methods:**

Studies eligible for the efficacy of adjuvant targeted therapy regimens in advanced or metastatic RCC published before December 2021 in PubMed, Embase, Cochrane Clinical Trials Database (CENTRAL), and Web of Science were searched for (1) patients with locally advanced renal cell carcinoma (RCC) who received adjuvant postoperative targeted therapy versus those not receiving active treatment; (2) primary endpoint outcomes of disease-free survival (DFS), overall survival (OS), and adverse events (AEs); and (3) design: randomized controlled trial (RCT) as inclusion criteria. Data on DFS and OS were extracted or recalculated by meta-analysis as hazard ratios (HRs), and AEs were compared using a dominance ratio (OR).

**Result:**

This systematic evaluation will provide evidence on the effectiveness and adverse effects of adjuvant targeted therapy in patients with advanced RCC. The results of meta-analysis showed that all of the three adjuvant targeted therapeutic drugs (sorafenib, sunitinib, and pazopanib) did not benefit from the adjuvant targeted therapy for DFS and OS and even increase the incidence of AEs compared to the placebo.

**Conclusions:**

The aim of this study was to summarize data on DFS, OS, and AEs in patients with advanced RCC treated with targeted therapies. The evidence provided by this systematic evaluation and meta-analysis will help guide clinical decision-making and provide insight into the future management of patients with advanced RCC.

## 1. Introduction

Renal cell carcinoma (RCC) accounts for 80-85% of all kidney cancers, and it is the most common and third most commonly diagnosed genitourinary malignancy [1, 2]. It usually occurs between the ages of 60 and 70 years and is most common in men [3]. Global incidence varies, with the highest incidence in developed countries such as North America and Europe, and incidence in Asia is now increasing yearly [4].

The management of RCC has changed dramatically in the last two decades. With little effective treatment options for the disease other than surgical resection, systemic treatment of RCC now includes a wealth of options, including inhibition of the vascular endothelial growth factor (VEGF) pathway via VEGFR-tyrosine kinase inhibitors (VEGF TKI) or the anti-VEGF antibody bevacizumab, mTOR pathway inhibition, and immune checkpoint inhibitors (ICI) [5, 6]. Recently, ICI-based combinations (either ICI-ICI or ICI-VEGF TKI) for the treatment of advanced RCC and today form the standard of care first-line therapy for patients with this disease have shown significant efficacy [7].

The article "The Efficacy of Adjuvant Targeted Therapy in Patients with Advanced Renal Cell Carcinoma: A Systematic Review and Meta-Analysis" was retracted in 2023. Reasons: unreliable results or conclusions; concerns about the data; concerns about the peer review; concerns about the citations.

Sorafenib is a multikinase inhibitor of tumor cell proliferation and angiogenesis; it has an effect on tumor cell proliferation and tumor angiogenesis and was originally identified as a Raf kinase inhibitor. It also inhibits vascular endothelial growth factor receptor (VEGFR) 1, 2, and 3; platelet-derived growth factor receptor *β* (PDGFR*β*); FMS-like tyrosine kinase 3 (Flt-3); c-Kit protein (c-Kit); and RET receptor tyrosine kinase [8–10].

Sunitinib, a vascular endothelial growth factor receptor tyrosine kinase inhibitor, is the standard of care in the first-line treatment of advanced RCC [11, 12]. In a large randomized phase 3 trial involving previously untreated patients, sunitinib had a median progression-free survival of 9.5 months, an objective remission rate of 25%, a median overall survival of 29.3 months, and haematological toxic effects [13].

Pazopanib, a polytyrosine kinase, was approved in the phase 3 PALETTE trial after failure of standard chemotherapy in patients with metastatic nonadipocytic RCC. Liposarcoma is included in this trial and further trials as there was still uncertainty about the role of pazopanib in liposarcoma at the time of designing this trial [14–16]. Pazopanib is now a first-line targeted therapy for advanced RCC [17].

The results were searched for articles on the efficacy and adverse effects of adjuvant targeted therapy with sorafenib, sunitinib, and pazopanib-targeted drugs in advanced or metastatic RCC for meta-analysis and systematic evaluation to guide clinical decision-making and provide insight into the future management of patients with advanced RCC.

## 2. Material and Methods

### 2.1. Literature Search Strategy

We conducted a comprehensive literature search to retrieve eligible studies published before December 2021 in the following electronic database of PubMed, Embase, Cochrane Clinical Trials Database (CENTRAL), and Web of Science and used the following keywords: “kidney” or “renal” and “cancer” or “tumor” or “carcinoma” or “neoplasm” and “adjuvant targeted therapy” or “adjuvant targeted treatment” or “targeted therapy.” Full-text reviews were performed if the abstracts were insufficient for determining if the studies met the inclusion or exclusion criteria. The reference lists of the retrieved articles and review articles were examined manually to identify further relevant studies not identified using the search strategy.

The article "The Efficacy of Adjuvant Targeted Therapy in Patients with Advanced Renal Cell Carcinoma: A Systematic Review and Meta-Analysis" was retracted in 2023. Reasons: unreliable results or conclusions; concerns about the data; concerns about the peer review; concerns about the citations.

### 2.2. Study Selection

The inclusion criteria were as follows: (1) patients receiving treatment adjuvant targeted therapy versus no active treatment after surgery among patients with locally advanced RCC; (2) primary endpoint outcome was disease-free survival (DFS), overall survival (OS), and adverse events (AEs); (3) design: randomized controlled trials (RCTs); and (4) only articles with full text available in English were selected. The exclusion criteria the reviewers agreed upon were as follows: (1) reviews, letters, or protocols; (2) duplicate articles; and (3) no sufficient related outcomes.

### 2.3. Data Extraction

Two reviewers (J Chen and B Zhao) independently extracted data based on predefined criteria, and any disagreements were resolved by consulting a third reviewer. Reviewers extracted the following data from each eligible study: first author's name, country of origin, year of publication, study design, characteristics of study patients (sample size, age, gender, and disease stage), treatment measures, and the results of primary outcomes (DFS, OS, and AEs).

### 2.4. Quality Assessment

All included documents were evaluated according to the Cochrane quality evaluation criteria: whether the study control adopts a random method; whether the study assignment is hidden; whether the evaluation of the outcome event adopts independent blind evaluation or identification; the completeness of the follow-up, whether to explain the number of people lost to follow-up and the reason; whether the study has intention analysis; and whether the studies are comparable.

### 2.5. Statistical Analysis

Meta analysis was performed by using Revman 5.4 (The Cochrane Collaboration, Oxford, UK) and STATA 14.0 (STATA Corp., College Station, TX, USA). Specifically, data for DFS and OS were extracted or recalculated as hazard ratio (HR), and odds ratios (OR) were used for comparison of AEs. Heterogeneity of the data was assessed using *I*^2^ values. If *P* < 0.05 or *I*^2^ > 50%, random effects model would be used for analysis; if *P* ≥ 0.05 and *I*^2^ ≤ 50%, fixed effects model would be used for analysis. We will conduct a sensitivity analysis by excluding merged studies one by one and observe whether the synthesis result changed significantly. Furthermore, funnel plot would be used to identify publication bias, *P* > 0.05 indicated that there was no publication bias.

The article "The Efficacy of Adjuvant Targeted Therapy in Patients with Advanced Renal Cell Carcinoma: A Systematic Review and Meta-Analysis" was retracted in 2023. Reasons: unreliable results or conclusions; concerns about the data; concerns about the peer review; concerns about the citations.

## 3. Results

### 3.1. Search Process

A total of 482 articles were identified by the screening electronic search strategy. After removal of duplicates, 368 articles were identified. After going through the titles and abstracts, 323 articles were excluded. After careful reading of full-text, 38 studies were further excluded because of the study design and insufficient data presented. Thus, 7 studies met the criteria for inclusion in the present meta-analysis [18–24]. The detailed search process was presented in Figure 1.

### 3.2. Characteristics of Included Studies

The baseline characteristics of the included studies were presented in Table 1. All the 7 studies were RCTs and were phase III clinical trials. A total of 8987 RCC patients were included. Adjuvant targeted therapeutic drugs included sunitinib, sorafenib, and pazopanib, of which 4 studies used sunitinib, 3 studies used sorafenib, and 2 studies used pazopanib. All were placebo-controlled studies. The countries where the trails were carried out included the United States and France.

### 3.3. Results of Quality Assessment

After identifying the reports, the abstracts and full texts were carefully read, and the publication's quality was screened and evaluated according to the Cochrane bias risk assessment. The quality evaluation table of literature was shown in Figure 2. One study could not download the basic information of patients, two studies lacked data of AEs, and one study only reported OS but not DFS.

### 3.4. Results of the Meta-Analysis for Outcomes

#### 3.4.1. Disease-Free Survival

Six literature studies reported DFS, and the results of heterogeneity test showed that there was no significant heterogeneity among the included studies (*I*^2^ = 5%, *P* = 0.39), so the fixed effects model was performed for pooled analysis. The overall HR was 0.92 (95% CI [0.85, 0.99], *P* = 0.04), suggesting that DFS in the intervention group was lower than that in the control group (Figure 3). Subgroup analysis were performed according to the different adjuvant targeted therapeutic drugs. The pooled HR of DFS in sorafenib group, sunitinib group, and pazopanib group were (HR = 0.97, 95% CI [0.85, 1.10], *P* = 0.64), (HR = 0.89, 95% CI [0.80, 1.00], *P* = 0.06), and (HR = 0.86, 95% CI [0.70, 1.06], *P* = 0.16), respectively. There was no significant difference in three groups, suggesting that each group did not benefit from the adjuvant targeted therapy for DFS. The result of sensitivity analysis showed that no independent study was an obvious source of heterogeneity, which is suggesting that the result was relatively reliable (Figure 4(a)).

The article "The Efficacy of Adjuvant Targeted Therapy in Patients with Advanced Renal Cell Carcinoma: A Systematic Review and Meta-Analysis" was retracted in 2023. Reasons: unreliable results or conclusions; concerns about the data; concerns about the peer review; concerns about the citations.

#### 3.4.2. Overall Survival

All the seven studies reported OS, and there was no significant heterogeneity among the included literatures (*I*^2^ = 0%, *P* = 0.70), so the fixed effects model was used for combined effect size analysis, and the results of meta-analysis showed that the pooled HR of OS was 0.99 (95% CI [0.90, 1.08], *P* = 0.75), indicating that there was no difference between the intervention group and the control group for OS (Figure 5). The pooled HR of OS in sorafenib group, sunitinib group, and pazopanib group were (HR = 0.97, 95% CI [0.84, 1.11], *P* = 0.63), (HR = 1.05, 95% CI [0.90, 1.23], *P* = 0.51), and (HR = 0.93, 95% CI [0.77, 111], *P* = 0.41), respectively. There were no significant difference in three groups, suggesting that adjuvant targeted therapy in each group did not improve OS after intervention. The sensitivity analysis showed that the result was not changed by omitting one study in each turn, indicating the result was robust (Figure 4(b)).

#### 3.4.3. AEs

Five literature studies reported on AEs caused by treatment. Due to the large amount of data, this study only analyzed high-grade AEs (grade ≥ 3). The main AEs caused by targeted therapy contained hypertension, rash, hand-foot syndrome, diarrhea, fatigue, neutropenia, nausea, mucositis, headache, vomiting, and decreased appetite. Compared with placebo, the differences in different types of AEs caused by adjuvant targeted therapy were shown in Table 2. The results showed that all the different types of AEs caused by targeted therapy were higher than those in the placebo group, especially hand-foot syndrome (OR = 26.29, 95% CI [16.72, 41.34]; *P* < 0.001), mucositis (OR = 16.07, 95% CI [5.85, 44.12]; *P* < 0.001), rash (OR = 15.38, 95% CI [8.00, 29.57]; *P* < 0.001), diarrhea (OR = 14.56, 95% CI [8.46, 25.05]; *P* < 0.001); and decreased appetite (OR = 11.56, 95% CI [2.73, 48.9]; *P* < 0.001).

### 3.5. Publication Bias

A funnel plot was performed to evaluate the publication bias. Two funnel plots were produced according the data of DFS and OS, and the plots showed some evidence of symmetry (Figure 6). The Egger's linear regression for quantitatively evaluating publication bias of outcomes was nonsignificant (DFS, *P* = 0.752; OS, *P* = 0.491), which suggested that no significant publication bias was existed in our meta-analysis.

## 4. Discussion

Most clinicians currently favor targeted therapy as the treatment option for patients with advanced RCC; however, the effectiveness of targeted therapy remains controversial. Many studies still suggest that targeted therapy is not effective in treating advanced cancer [25–27].

We searched and screened the relevant RCT literature for targeted therapies for RCC and performed DFS, OS, and AEs analyses with similar no benefit findings: the DFS: meta-analyses for the sorafenib, sunitinib, and pazopanib groups were [HR = 0.97, 95% CI (0.85, 1.10), *P* = 0.64], [HR = 0.89, 95% CI (0.80, 1.00), *P* = 0.06], and [HR = 0.86, 95% CI (0.70, 1.06), *P* = 0.16], respectively; OS: [HR = 0.97, 95% CI (0.84, 1.11), *P* = 0.63], [HR = 1.05, 95% CI (0.90, 1.23), *P* = 0.51], and [HR = 0.93, 95% CI (0.77, 1.11), *P* = 0.41] for the sorafenib, sunitinib, and pazopanib groups, respectively; and AEs suggested an increase in adverse effects in patients with RCC treated with targeted drugs, especially hand-foot syndrome [OR = 26.29, 95% CI (16.72, 41.34); *P* < 0.001], mucositis [OR = 16.07, 95% CI (5.85, 44.12); *P* < 0.001], rash [OR = 15.38, 95% CI (8.00, 29.57); *P* < 0.001], diarrhea [OR = 14.56, 95% CI (8.46, 25.05); *P* < 0.001], and decreased appetite [OR = 11.56, 95% CI (2.73, 48.9); *P* < 0.001].

The article "The Efficacy of Adjuvant Targeted Therapy in Patients with Advanced Renal Cell Carcinoma: A Systematic Review and Meta-Analysis" was retracted in 2023. Reasons: unreliable results or conclusions; concerns about the data; concerns about the peer review; concerns about the citations.

There are many controversies surrounding new treatment options such as targeted therapies, and some studies have shown that targeted therapies do have benefits [28–30]. However, there are still many clinical issues that need to be addressed; more tests may need to be added to further screen suitable populations for more precise targeted therapies, or the dose of targeted drugs may need to be more tightly controlled to avoid adverse effects. The dose of targeted drugs may need to be more tightly controlled to avoid adverse effects.

## Figures and Tables

**Figure 1:** Flow diagram of study selection in the systematic review and meta-analysis.

**Figure 2:** Risk of bias in included studies. (a) Bias assessment summary. (b) Risk of bias for each study. Green: low risk; yellow: unclear; and red: high risk.

**Figure 3:** Forest plot for DFS between intervention group and control group.

**Figure 4:** Sensitivity analysis of (a) DFS and (b) OS.

**Figure 5:** Forest plot for OS between intervention group and control group.

**Figure 6:** Funnel plot for potential publication bias. (a) DFS; (b) OS.

**Table 1:** Baseline characteristics of the studies included in this meta-analysis.

Study	Study design	Country	Trial phase	Patients stage	Treatment		No. of patients		Age^a^		Gender (M/F)	
					Intervention	Control	Intervention	Control	Intervention	Control	Intervention	Control
Ravaud 2016	RCT	France	III	Locoregional, high-risk clear-cell RCC	Sunitinib 50 mg per day	Placebo	309	306	57 (25–83)	58 (21–82)	222/87	229/77
Haas 2016	RCT	USA	III	High-risk, non-metastatic RCC	Sunitinib 50 mg per day	Placebo	647	647	56 (49–64)	57 (49–64)	429/218	443/204
					Sorafenib 400 mg twice per day	Placebo	649	647	55 (48–63)	57 (49–64)	437/212	443/204
Motzer 2017	RCT	USA	III	pT2 (high grade) or ≥pT3, including N1, clear cell RCC	Pazopanib, starting 600 mg/d for 1 yr, with optional dose escalation to 800 mg/d after 8–12 wk	Placebo	571	564	58 (22-83)	58 (21–82)	398/173	400/164
Haas 2017	RCT	USA	III	High-risk (pT3, pT4, node-positive) clear RCC	Sunitinib 50 mg per day	Placebo	358	356	59 (31–83)	58 (19–83)	243/115	254/102
					Sorafenib 400 mg per day	Placebo	355	356	56 (20–84)	58 (19–83)	248/107	254/102
Motzer 2018	RCT	USA	III	Nonmetastatic locoregional RCC defined as T3 or T4	Sunitinib 50 mg per day	Placebo	309	306	57 (49–64)	58 (51–66)	222/87	229/77
Motzer 2021	RCT	USA	III	Stage T1/T2, T3, T4	Pazopanib, starting 800 mg/d, reduced to 600 mg/d following a blinded safety review	Placebo	769	769	NR	NR	NR	NR
Eisen 2020	RCT	USA	III	pT1, pT2, pT3a-4	Sorafenib 400 mg once-twice daily	Placebo	639	430	57.97 ± 10.86	58.43 ± 10.35	458/181	306/124

RCT: randomized controlled trials; RCC: renal cell carcinoma; NR: not reported. ^a^Values were expressed as mean ± standard deviation or median (range).

The article "The Efficacy of Adjuvant Targeted Therapy in Patients with Advanced Renal Cell Carcinoma: A Systematic Review and Meta-Analysis" was retracted in 2023. Reasons: unreliable results or conclusions; concerns about the data; concerns about the peer review; concerns about the citations.

**Table 2:** The difference of AEs between intervention group and control group.

Adverse events	Subgroup	*n*	Subgroup OR (95% CI)	Subgroup *P* value	Pooled OR (95% CI)	Pooled *P* value
Hypertension	Sorafenib	3	2.35 (0.71, 7.82)	0.160	3.47 (2.10, 5.74)	<0.001
	Sunitinib	3	4.69 (3.21, 6.86)	<0.001		
	Pazopanib	1	4.65 (3.17, 6.83)	<0.001		
Rash	Sorafenib	3	28.51 (11.11, 73.15)	<0.001	15.38 (8.00, 29.57)	<0.001
	Sunitinib	3	4.62 (1.66, 12.86)	0.003		
	Pazopanib	1	2.95 (0.12, 72.63)	0.510		
Diarrhea	Sorafenib	3	14.84 (6.02, 36.59)	<0.001	14.56 (8.46, 25.05)	<0.001
	Sunitinib	3	18.03 (7.30, 44.52)	<0.001		
	Pazopanib	1	9.93 (3.52, 28.01)	<0.001		
Hand-foot syndrome	Sorafenib	3	41.82 (20.81, 84.02)	<0.001	26.29 (16.72, 41.34)	<0.001
	Sunitinib	3	16.33 (8.80, 30.29)	<0.001		
	Pazopanib	1	23.04 (1.35, 391.95)	0.030		
Nausea	Sorafenib	3	3.01 (0.85, 10.68)	0.090	8.08 (3.37, 19.35)	<0.001
	Sunitinib	3	17.41 (4.18, 72.53)	<0.001		
	Pazopanib	1	4.93 (0.24, 102.91)	0.300		
Fatigue	Sorafenib	3	2.24 (1.39, 3.62)	0.001	4.06 (2.98, 5.54)	<0.001
	Sunitinib	3	5.94 (3.90, 9.05)	<0.001		
	Pazopanib	NR	—	—		
Vomiting	Sorafenib	2	2.68 (0.71, 10.12)	0.150	4.50 (2.04, 9.93)	<0.001
	Sunitinib	3	7.10 (2.31, 21.81)	<0.001		
	Pazopanib	1	0.98 (0.06, 15.74)	0.990		
Mucositis	Sorafenib	2	11.16 (2.09, 59.45)	0.005	16.07 (5.85, 44.12)	<0.001
	Sunitinib	3	22.71 (5.50, 93.77)	<0.001		
	Pazopanib	1	4.93 (0.24, 102.91)	0.300		
Neutropenia	Sorafenib	2	2.44 (1.27, 4.70)	0.008	2.99 (1.92, 4.67)	<0.001
	Sunitinib	3	3.52 (1.91, 6.46)	<0.001		
	Pazopanib	NR	—	—		
Headache	Sorafenib	1	3.02 (1.79, 5.10)	<0.001	2.72 (1.89, 3.93)	<0.001
	Sunitinib	2	2.48 (1.46, 4.20)	<0.001		
	Pazopanib	1	1.97 (0.18, 21.77)	0.580		
Decreased appetite	Sorafenib	1	11.05 (0.61, 200.31)	0.100	11.56 (2.73, 48.9)	<0.001
	Sunitinib	2	15.18 (2.01, 114.88)	0.008		
	Pazopanib	1	4.93 (0.24, 102.91)	0.300		

OR: odds ratio; CI: confidence interval; NR: not reported.

The article "The Efficacy of Adjuvant Targeted Therapy in Patients with Advanced Renal Cell Carcinoma: A Systematic Review and Meta-Analysis" was retracted in 2023. Reasons: unreliable results or conclusions; concerns about the data; concerns about the peer review; concerns about the citations.

## Data Availability

No data were used to support this study.
